The article "Effect of Perioperative Comprehensive Nursing Intervention on the Rehabilitation Effect of Radiofrequency Ablation for Patients with Hypertrophic Obstructive Cardiomyopathy" was published in 2022. Journal: Contrast Media Mol Imaging.

# Effect of Perioperative Comprehensive Nursing Intervention on the Rehabilitation Effect of Radiofrequency Ablation for Patients with Hypertrophic Obstructive Cardiomyopathy

**DOI:** 10.1155/2022/6436073

**Published:** 2022-08-11

**Authors:** Xiaoping Xiang, Yanru Chen, Lijun Dai

**Affiliations:** Imaging Nuclear Medicine Interventional Nursing Unit, The Second Affiliated Hospital and Yuying Children's Hospital, Wenzhou Medical University, Wenzhou 325000, Zhejiang, China

## Abstract

**Objective:**

The aim of the study was to determine standardized perioperative nursing for radiofrequency ablation of hypertrophic obstructive cardiomyopathy under the guidance of intracardiac ultrasound, which can improve the quality of nursing.

**Methods:**

From January 2020 to November 2021, 40 patients with hypertrophic obstructive cardiomyopathy who underwent radiofrequency ablation under the guidance of intracardiac ultrasound in our hospital were selected. Patients were grouped according to their use of standardized perioperative nursing. Patients from both cohorts were compared for negative emotions, depression, and anxiety at the baseline and at month 2.

**Results:**

In general, there were no differences between the two groups (*P* > 0.05). At admission, the Self-rating Depression Scale (SDS) and Self-rating Anxiety Scale (SAS) scores of these two groups showed no differences (*P* > 0.05). Following nursing, the scores of the two groups dropped significantly, with the control group scoring much lower than the experimental group. Among the experimental group, the satisfaction rate was 100.00%, whereas the control group had an 85.00% satisfaction rate (*P* < 0.05). Following nursing, the scores of the two groups dropped significantly, with the control group scoring much lower than the experimental group.

**Conclusions:**

To sum up, perioperative comprehensive nursing intervention during surgical treatment can quickly alleviate patients' clinical symptoms, reduce complications, damage to patients' body, reduce patients' pain, relieve patients' anxiety and depression, and improve overall sleep quality and clinical nursing satisfaction.

## 1. Introduction

Hypertrophic obstructive cardiomyopathy is a kind of cardiomyopathy characterized by left ventricular outflow tract obstruction and uneven hypertrophy of the ventricular septum [1, 2]. The global adult incidence rate is 0.02% ∼ 0.23%, and in China, it is about 0.08% [3]. Hypertrophic obstructive cardiomyopathy is characterized by regional asymmetric myocardial hypertrophy, which most often occurs under the aortic valve [4, 5]. Left ventricular outflow tract obstruction can be detected by echocardiography, resulting in chest pain, dyspnea, and sudden death [6]. It is difficult for most patients to effectively improve or control their symptoms through drug treatment [6, 7]. Surgical thoracotomy is considered to be the “gold standard” of nondrug treatment. However, it has some shortcomings, such as great trauma and slow recovery of patients [7]. Therefore, alcohol ventricular septal ablation has become an option, but about 5–15% of patients cannot complete the operation due to lack of the appropriate ventricular septal artery or anatomical reasons [8–10]. In addition, more than 30% of patients will develop atrioventricular block, which greatly increases the risk of sudden cardiac death [11]. With the development of medical technology and instruments, radiofrequency ablation of hypertrophic obstructive cardiomyopathy under the guidance of intracardiac ultrasound has been gradually applied in clinics in recent years, which can accurately guide the fixed-point and quantitative ablation of the obstruction so as to make local myocardial necrosis and form scar tissue, reduce the obstruction of the outflow tract, and improve the clinical symptoms of patients [12–14].

The article "Effect of Perioperative Comprehensive Nursing Intervention on the Rehabilitation Effect of Radiofrequency Ablation for Patients with Hypertrophic Obstructive Cardiomyopathy" was published in 2022. Journal: Contrast Media Mol Imaging.

Cardiovascular interventional surgery is welcomed and accepted by the majority of patients because of its advantages of small trauma, rapid postoperative recovery, and low hospitalization expenses [14–16]. The success of interventional therapy is inseparable from the close cooperation of nursing staff [17]. Whether in terms of preoperative publicity and education, venous access preparation, intraoperative attention to patients, cooperation with doctors, and prevention of postoperative complications, if the nursing work mode is not standardized, it is bound to affect the safety of operation and the rehabilitation of patients. Radiofrequency ablation of hypertrophic obstructive cardiomyopathy under the guidance of intracardiac ultrasound is a new and sophisticated operation in recent years [18]. At present, nurses lack a systematic understanding of the operation, the preparation of intraoperative instruments, and the prevention of surgical complications [18–20].

Therefore, we hypothesized that standardized perioperative nursing for radiofrequency ablation of hypertrophic obstructive cardiomyopathy under the guidance of intracardiac ultrasound can improve the quality of nursing [21], further reduce the incidence of complications, and play an important clinical significance for the follow-up treatment and rehabilitation of patients.

## 2. Methods

### 2.1. Participants

From January 2020 to November 2021, 40 patients with hypertrophic obstructive cardiomyopathy who underwent radiofrequency ablation under the guidance of intracardiac ultrasound in our hospital were selected. After the patient is admitted, we inform the nursing situation. Patients can choose what type of care they want. The former was given routine nursing, while the latter was given perioperative standardized nursing. This study was approved by the medical ethics association of our college, and all patients signed informed consent. Inclusion criteria were as follows: (1) patients with previous symptoms such as chest pain, exertional dyspnea, syncope, and cardiac insufficiency; (2) relevant valve diseases were excluded, and patients met the diagnostic criteria of echocardiography: ventricular septal thickness >15 mm and ventricular septal thickness/left ventricular posterior wall ≥1.3; (3) patients with the left ventricular outflow tract pressure difference >50 mmHg at rest or ≥70 mmHg under stress; (4) patients unable to receive medication or medication cannot improve symptoms. Exclusion criteria were as follows: (1) patients with the thickness of the ventricular septum did not meet the diagnostic criteria (<15 mm); (2) patients with the ventricular septal thickness >15 mm, while those with the left ventricular outflow tract pressure difference did not meet the diagnostic criteria; (3) those with concomitant cardiac surgical diseases such as multibranch coronary artery disease or severe mitral valve disease; (4) those with other organ dysfunction combined with liver and kidney function and who cannot tolerate surgery.

The article "Effect of Perioperative Comprehensive Nursing Intervention on the Rehabilitation Effect of Radiofrequency Ablation for Patients with Hypertrophic Obstructive Cardiomyopathy" was published in 2022. Journal: Contrast Media Mol Imaging.

### 2.2. Nursing Care Delivery Strategies

The control group received conventional nursing care. Basic nursing: through the self-made evaluation form, we observe the patient's previous medical history, whether there is heparin resistance, whether the preoperative examination is perfect, in addition to the routine preoperative items (such as blood routine, blood biochemistry, bleeding and coagulation, and chest), especially we record the left ventricular outflow tract pressure difference under resting or excitation, and whether the electrocardiogram(ECG) scan indicates conduction block. Specialized nursing: whether the surgical clothes are appropriate, whether the electrode parts on the body surface are clean, and whether the venous pathway is unobstructed. For patients with poor venous conditions, two pathways or deep venous pathways can be prepared. We should prepare the required catheter, check the validity period and performance of the equipment to ensure that it is in good condition, communicate with each other about the items that may be needed during the operation and the habits of the operator, be aware of them, and check the good preparation in time. Psychological nursing: we actively communicate with patients, obtain full trust, appease emotions, and introduce the operation process and points for attention during operation. Most patients have different degrees of anxiety and tension in the face of surgical treatment, and nurses should dredge them in time and introduce patients with disease-related knowledge, such as surgical purpose and process and precautions after operation so as to increase their understanding of surgical treatment and improve their nursing compliance. Perioperative standardized intraoperative nursing: we check the completion of nursing observation indexes one by one through the self-made intraoperative nursing standardized completion table. a. We place the patient in a supine position and ask them to take a comfortable position. *b*. Due to the long operation time, a simple artificial urine bag is retained during the operation to avoid polluting the operating table and wetting the caudal sacral part so as to improve comfort; *c*. We protect our hands from slipping and observe the preparation of drugs and articles through the scale. Intraoperative complications are observed. We communicate with patients during the operation, comfort them, and accompany them beside the bed when necessary to reduce anxiety. 3. Standardized postoperative care during the perioperative period: after the operation, the femoral artery and vein puncture points are pressurized and bandaged, 2 kg sandbags compress the wound, four people across the bed notify the ward, follow, and monitor the critically ill patients who may have cardiac events on the way back to the ward, and we prepare corresponding first-aid drugs and carry simple breathing balloons so that accidents can be handled in time. Guide the change in patients' body position, we strengthen psychological and life care while breaking the limbs, massage and break the limbs to promote blood circulation, guide the methods of urination and defecation on the bed again, strengthen the inspection of the puncture site, keep the puncture site clean, and dry and prevent infection. For those who are nervous and sensitive to pain, we prevent the occurrence of the vagal reflex and prepare first-aid drugs.

The article "Effect of Perioperative Comprehensive Nursing Intervention on the Rehabilitation Effect of Radiofrequency Ablation for Patients with Hypertrophic Obstructive Cardiomyopathy" was published in 2022. Journal: Contrast Media Mol Imaging.

### 2.3. Observation Index

Patients from both cohorts were compared for negative emotions, depression, and anxiety at the baseline and at month 2.

#### 2.3.1. Emotional Status

To evaluate depression, we used the Self-rating Depression Scale (SDS). The Self-rating Anxiety Scale (SAS) was used to measure anxiety levels of patients. Both scales have scores ranging from 1 to 4. The scores from each scale were multiplied by 1.25. The scores of 50 or more on the SAS indicate anxiety, and the scores of more than 53 on the SDS indicate sustained depression. Psychological morbidity is associated with higher scores on these scales.

#### 2.3.2. Satisfaction

After consulting the literature and experts' discussion, we designed patients' follow-up satisfaction. The patients in the patient satisfaction survey were asked to rate the nursing they received based on their feelings regarding nurses' attitude, their operating skills, their mastery of knowledge, and their comfort level. In the survey, there were 25 questions, each with four options, namely, dissatisfied, partially satisfied, satisfied, and highly satisfied on a 1 to 4 scale.

### 2.4. Statistical Analysis

Analyses of this research were conducted using *R* software. The measurement data are expressed as the mean ± SD, and the counting data are displayed in percentage. To measure the differences between the two cohorts, the chi-square test or Student's *t*-test was utilized.

## 3. Results

### 3.1. Subject Characteristics

As shown in Table 1, the baseline characteristics of the cohorts are described. In general, there were no differences between the two groups (*P* > 0.05).

### 3.2. Emotional Status

At admission, the SAS and SDS scores of these two groups showed no differences (*P* > 0.05, Table 2). Following nursing, the scores of the two groups dropped significantly, with the control group scoring much lower than the experimental group.

### 3.3. Satisfaction

The satisfaction of nurses was compared. Among the experimental group, the satisfaction rate was 100.00%, whereas the control group had an 85.00% satisfaction rate (*P* < 0.05, Table 3).

## 4. Discussion

Alcohol ventricular septal ablation is a new and effective method for the treatment of hypertrophic obstructive cardiomyopathy [9, 15]. It is also the best treatment at present. Compared with surgery, alcohol ventricular septal ablation has the same effect, but it has the advantages of convenience, practicality, economy, and less trauma [10, 13]. However, the operation is technically difficult and has many and serious postoperative complications [22]. At present, there are still not many hospitals that can carry out this kind of operation. The success and postoperative effect of the operation depend on the technology of medical staff, the psychological quality of patients, and good living habits [23, 24].

Hypertrophic obstructive cardiomyopathy has a high incidence rate in young adults, with more males than females [25, 26]. Due to the long-term repeated chest pain with syncope, the physical and mental burden of patients is very heavy. They often show anxiety and fear before operation, which reduces the pain threshold, aggravates the chest pain during operation, and greatly increases the incidence of vagal reflex and arrhythmia. Therefore, it is very important to stabilize the anxiety and fear of patients. After operation, close ECG monitoring and condition observation are needed, which requires nurses to master the operation principle, understand ECG, and quickly identify the condition and then take standardized postoperative nursing to ensure the life safety of patients. In order to improve the operation efficiency and relieve the discomfort of patients in time, it is necessary to provide corresponding nursing measures for patients [27]. Perioperative comprehensive nursing is a systematic nursing operation, which is of great significance to the rehabilitation of patients.

The article "Effect of Perioperative Comprehensive Nursing Intervention on the Rehabilitation Effect of Radiofrequency Ablation for Patients with Hypertrophic Obstructive Cardiomyopathy" was published in 2022. Journal: Contrast Media Mol Imaging.

Through this study, it can be concluded that before nursing, the patients in the two groups had heavy anxiety and depression psychology, the degree of pain was heavy, and the difference was not obvious. After nursing, the anxiety and depression psychology of the observation group were significantly reduced, and the pain was significantly improved. Before nursing, the patients in the two groups had poor sleep quality, and there was no significant difference between them. After nursing, the improvement effect of the sleep quality on the observation group was more significant than that on the control group. The satisfaction and recognition of nursing in the experiment group (100%) were significantly higher than those in the control group (82%). It can be seen that compared with the routine perioperative nursing operation, the effect of the perioperative comprehensive nursing intervention is more significant, which can quickly alleviate the discomfort of patients, accelerate the speed of postoperative rehabilitation, and improve the prognosis of patients [28]. The perioperative comprehensive nursing intervention is a systematic nursing operation. The nursing content starts before the patient receives the operation, and the preoperative preparatory nursing content is performed to make the patient physically and mentally ready for the operation and adjust their own state. The nursing cooperation of nursing staff during the operation can accelerate the operation speed, effectively prevent the occurrence of adverse reactions of patients, and ensure the smooth operation. The postoperative nursing operation can provide effective nursing content according to the patient's surgical operation so as to speed up the patient's postoperative recovery, improve the patient's symptoms, and improve the patient's prognosis.

Overall, the effect of the perioperative comprehensive nursing intervention is ideal. To sum up, providing the perioperative comprehensive nursing intervention during surgical treatment can quickly alleviate patients' clinical symptoms, reduce complications, damage to patients' body, reduce patients' pain, relieve patients' anxiety and depression, improve overall sleep quality and clinical nursing satisfaction, and improve patients' prognosis.

The article "Effect of Perioperative Comprehensive Nursing Intervention on the Rehabilitation Effect of Radiofrequency Ablation for Patients with Hypertrophic Obstructive Cardiomyopathy" was published in 2022. Journal: Contrast Media Mol Imaging.

## Figures and Tables

**Table 1:** Baseline characteristics.

	Control group	Experimental group	*P*
*N*	20	20	
Age, years	61.3 ± 10.4	64.4 ± 12.6	0.81

Sex, *n* (%)			0.73
Male	13 (65.0%)	14 (70.0%)	
Female	7 (35.0%)	6 (30.0%)	

BMI, kg/m^2^	24.5 ± 3.2	26.4 ± 3.5	0.091

*Treatment, n (%)*			
*β*-Blocker	14 (70.0%)	14 (70.0%)	1.00
ACEI	6 (30.0%)	7 (35.0%)	0.73
Calcium antagonist	7 (35.0%)	6 (30.0%)	0.73

*NYHA, n (%)*			1.00
III	19 (95%)	19 (95%)	
IV	1 (5%)	1 (5%)	

BMI: body mass index, ACEI: angiotensin-converting enzyme inhibitor, NYHA: New York Heart Function Assessment.

**Table 2:** SAS and SDS patients in the control group and the experimental group.

	Control group	Experimental group	*P* value
*SAS*			
0	68.8 ± 2.4	68.0 ± 2.4	0.31
2 months	50.0 ± 3.5	39.4 ± 9.3	<0.001

*SDS score*			
0	61.7 ± 10.2	66.5 ± 6.7	0.12
2 months	44.0 ± 10.4	33.1 ± 12.9	<0.001

**Table 3:** Nursing satisfaction of patients in the control group and experimental group.

	Control group	Experimental group	*P*-value
Satisfaction (%)	85.6 ± 17.9	100.0 ± 0.0	<0.001

SAS: Self-rating Anxiety Scale, SDS: Self-rating Depression Scale.

## Data Availability

The data supporting this study are available from the corresponding author upon request.
